# LNCRNA XIST Inhibits miR-377-3p to Hinder Th17 Cell Differentiation through Upregulating ETS1

**DOI:** 10.1155/2022/6545834

**Published:** 2022-06-14

**Authors:** Chen Yao, Chao Li, Zhijia Liu, Li Xiao, Hongwei Bai, Bingyi Shi

**Affiliations:** ^1^Beijing IROT Key Laboratory, The 8th Medical Center of Chinese PLA General Hospital, 100091 Beijing City, China; ^2^Department of Urology, The 8th Medical Center of Chinese PLA General Hospital, 100091 Beijing City, China

## Abstract

**Background:**

Th17 cell differentiation is involved in the development and progression of many diseases, such as rheumatoid arthritis and systemic lupus erythematosus. Present study mainly focused on the role of LINC-XIST in Th17 cell differentiation.

**Methods:**

The naïve CD4+ T cells were isolated from human whole blood. Cells were cultured under Th17 cell-polarizing condition for 6 days. The expression of LINC-XIST and miR-153-3p was measured by qPCR. The relationship between LINC-XIST, miR-153-3p, and ETS1 was predicted by TargetScan website and authenticated by luciferase reporter assay. ELISA assays were conducted to evaluate the IL-17 concentration. Western blot was utilized to measure the protein expression of ETS1. Th17 cell frequency was examined by flow cytometry.

**Results:**

The expression of XIST markedly decreased and miR-153-3p expression markedly increased with Th17 cell differentiation. The mRNA expression of IL-17, IL-17 concentration, and Th17 cell frequency were observably decreased in overexpressed LINC-XIST group. Luciferase reporter assay authenticated that miR-153-5p was directly regulated by LINC-XIST. miR-153-3p inhibitor observably decreased IL-17 concentration, mRNA expression of IL-17, and Th17 cell frequency while si-XIST reversed this impact. ETS1 was confirmed to be regulated by miR-153-5p via luciferase reporter assay. In addition, ETS1 markedly decreased IL-17 mRNA expression, IL-17 concentration, and Th17 cell frequency while miR-153-5p mimic reversed this impact.

**Conclusion:**

LNCRNA XIST inhibited miR-377-3p to hinder Th17 cell differentiation through upregulating ETS1.

## 1. Introduction

T lymphocytes (T cells) are the main components of lymphocytes, which mainly perform specific cellular immunity, which have an essential role in clearing pathogens and tumor cells and maintaining immune homeostasis [1]. T cells develop and mature in the thymus. When the body is stimulated by external antigen, T cells can differentiate to different cells like Th1, Th2, Th17, and Treg cells to participate in the body immune response [2]. Th17 cells can secrete IL-17, which could clear foreign pathogens and induce tissue inflammatory response. In the experiment of inducing T cell differentiation in vitro, TGF-*β* and IL-6 can induce the differentiation of Th17 cells and inhibit the differentiation of regulatory T cells (Treg cells) [3]. IL-21 and TGF-*β* can induce the expression of IL-23 receptor, promote Th17 cells differentiation, and inhibit the differentiation of Treg cells [4]. Th17 cell differentiation was reported to be regulated by non-coding RNA.

Long non-coding RNAs (LINC RNAs) are a class of non-coding RNA molecules with a length of more than 200 nucleotides, which are essential in cell growth, inflammatory response, and tumorigenesis [5]. LINC RNA can play its biological functions through a variety of mechanisms, such as mediating transcriptional regulation, controlling protein transport in the nucleus, regulating RNA stability, participating in chromatin remodeling, and so on [6]. Although most research on LINC RNA is in tumor, the research on LNC RNAs has also made significant progress in the field of immunology. The study reported that 1524 LINC RNAs were identified in 42 T cell subsets, which are located in the region rich in protein coding genes with immune regulation function [7]. LINC RNA could regulate the differentiation and balance of Treg and Th17 cells and also regulate the differentiation of Th1/Th2. Therefore, studying the role of XIST in Th17 cell differentiation and its specific mechanism is important, which can provide new solutions for the treatment of autoimmune diseases, infections, tumors, etc.

LINC RNA can be used as competitive endogenous RNAs to regulate mRNA by binding with miRNA as a molecular sponge. MicroRNA (miRNA) is a kind of non-coding small molecule RNA, which exists stably in various body fluids of human body and participates in the process of cell differentiation, proliferation, and apoptosis [8, 9]. Various miRNAs can regulate the differentiation of T cells, affect the function of various differentiated types of T cells and the secretion of related cytokines, and then participate in various pathophysiological processes in human body [10–12]. Recently, miRNA in body fluids has been reported as a new type of disease biomarker and shows promising applications. The differentiation of Th17 cells decreased after transfection with miR-301a-3p, which targeted PELI1 [10]. miR-155 targeted SOCS1 to promote Th17 cell differentiation and IL-17A production [11].

The present study aimed to explore the regulatory effect and mechanism of XIST on Th17 cell differentiation.

## 2. Materials and Methods

### 2.1. Isolation of Naïve CD4+ T Cells and Th17 Differentiation

The naïve CD4+ T cells were isolated from human whole blood via isolation kit. These cells were stimulated by 5 *μ*g/ml anti-CD3 antibody (R&D Systems) at 2–8°C. Then, cells were cultured under Th17 cell-polarizing condition using the CellXVivo Human Th17 Cell Differentiation Kit (R&D Systems) at 37°C in a humidified atmosphere containing 5% CO2 for 6 days. MiR-153-5p mimic and inhibitor expression vectors were synthesized by GenePharma. LINC-XIST expressing DNA fragments were cloned to the pcDNA3.1 vector for overexpression and a siRNA specific for XIST (si-XIST) was purchased from GenePharma.

### 2.2. RNA Isolation and Quantitative Real-Time PCR Analysis

Total RNA was separately extracted using the Trizol extraction reagent. The extracted total RNA was reverse transcribed to cDNA. RT-PCR was conducted according to the qPCR kit. Relative expression of XIST, miR-153-5p, and ETS1 was analyzed using the 2^−ΔΔ*Ct*^ method.

### 2.3. ELISA Assay

Culture supernatant was obtained to detect IL-17 concentration via ELISA assay according to the manufacturer's protocols.

### 2.4. Western Blot

Total protein from each group was extracted using RIPA lysate. SDS-PAGE was performed after detection of protein concentration. The membranes were transferred to methanol-activated PVDF membranes and blocked with 5% skim milk for 1 h at room temperature. Then, they were incubated with primary antibodies at 4°C overnight and washed three times with TBST. Then, they were incubated with goat anti-rabbit secondary antibody at room temperature for 2 h and washed three times with TBST and finally colored with an ECL chemiluminometer.

### 2.5. Flow Cytometry

Cells were resuspended with 50 *μ*L PBS and added with 10 *μ*L CD4-FITC antibody and incubated at 4°C for 30 min. After washing with 3 ml PBS and centrifugating at 1500 r/min for 10 min, the supernatant was discarded. Suspension was added with 250 mL Fix&Perm and incubated at room temperature for 20 min and washed again. Suspension was added with 100 mL Fix&Perm and PE-IL-17A and incubated without light 4°C for 30 min and washed again. Cells were resuspended in PBS and measured on the machine.

### 2.6. Luciferase Reporter Assay

We inserted the wild-type (WT) or mutant (MUT) XIST and ETS1 binding site in 3′UTR into the pGL3 vector (Promega, USA). 100 ng of the indicated luciferase reporter vector was co-transfected into HEK293T cells with 50 nM miR-153-3p or miR-NC by Lipofectamine 2000 (Invitrogen, USA). Then, the luciferase activity was detected after transfection for 48 h.

### 2.7. Statistical Analysis

Data were analyzed via SPSS.25. Differences of groups were compared using one-way analysis of variance (ANOVA). *P* values less than 0.05 were considered statistically significant.

## 3. Results

### 3.1. The Expression of LINC-XIST Decreased with Th17 Cell Differentiation

To detect the degree of differentiation of Th17 cells, we measured the concentration of IL-17 by ELISA. The concentration of IL-17 increased obviously with the increase of incubation time (Figure 1(a)). The expression of XIST obviously decreased with the increase of incubation time (Figure 1(b)). The expression of miR-153-3p increased obviously with the increase of incubation time (Figure 1(c)).

### 3.2. XIST Inhibited Th17 Cell Differentiation

XIST expression was observably increased after pcDNA-LINC-XIST transfection (Figure 2(a)). LINC-XIST observably decreased the mRNA expression of IL-17 (Figure 2(b)). LINC-XIST observably decreased the IL-17 concentration (Figure 2(c)). LINC-XIST observably decreased Th17 cell frequency (Figures 2(d) and 2(e)).

### 3.3. miR-153-5p Was Directly Regulated by XIST

It was predicted by TargetScan that miR-153-5p may be regulated by XIST (Figure 3(a)). miR-153-5p observably inhibited luciferase activity of XIST-WT while it did not change luciferase activity of XIST-MUT (Figure 3(b)). The expression of miR-153-5p was observably decreased in LINC-XIST group (Figure 3(c)).

### 3.4. XIST Reversed the Promoting Effect of miR-153-5p on Th17 Cell Differentiation

miR-153-3p inhibitor obviously decreased miR-153-3p expression while si-XIST observably inhibited miR-153-3p expression (Figure 4(a)). miR-153-3p inhibitor observably suppressed IL-17 mRNA expression (Figure 4(b)) and IL-17 concentration (Figure 4(c)) while si-XIST reversed this impact. miR-153-3p inhibitor observably suppressed Th17 cell frequency while si-XIST reversed this impact (Figures 4(d) and 4(e)).

### 3.5. miR-153-5p Directly Downregulated ETS1 Expression

It was predicted by TargetScan that ETS1 may be regulated by miR-153-5p (Figure 5(a)). miR-153-5p observably inhibited luciferase activity of ETS1-WT while it did not change luciferase activity of ETS1-MUT (Figure 5(b)). The protein expression of ETS1 was observably decreased in miR-153-5p group (Figures 5(c) and 5(d)).

### 3.6. miR-153-5p Reversed the Inhibiting Effect of ETS1 on Th17 Cell Differentiation

Firstly, result of qPCR indicated that ETS1 obviously increased ETS1 mRNA expression while miR-153-5p mimic observably decreased ETS1 mRNA expression (Figure 6(a)). ETS1 observably suppressed IL-17 mRNA expression (Figure 6(b)) and IL-17 concentration (Figure 6(c)) while miR-153-5p mimic reversed this impact. ETS1 observably suppressed Th17 cell frequency while miR-153-5p mimic reversed this impact (Figures 6(d) and 6(e)).

## 4. Discussion

Lymphocytes are important immune cells in the human body, including T cells, B cells, and NK cells that mediate cellular, humoral, and natural immunity, respectively [1]. T cells are considered the most abundant and functional class of cells in lymphocytes. They come from bone marrow lymphoid stem cells and differentiate, develop, and mature within the thymus, accounting for 65.0%–75.0% of peripheral lymphocytes [2]. Th17 cells are novel CD4+ effector T cells differentiated from naïve T cell precursors. Th17 cell has its independent differentiation and developmental regulatory mechanisms and produces IL-17 [13]. It is essential in autoimmune, infectious diseases and transplantation rejection and is an important component and mechanism of T cell immune response.

LINC-MAF-4 inhibited the expression of transcription factor MAF in Th2 cells and promoted the Th1 cell differentiation [14]. LncRNA RMRP is located in the nucleus of Th17 cells and promoted Th17 cell differentiation. Knockout of LincRNA RMRP could lead to impaired cytokine secretion in Th17 cells [15]. The present study demonstrated that the expression of LINC-XIST obviously decreased with Th17 cell differentiation and LINC-XIST observably inhibited IL-17 concentration, mRNA expression of IL-17, and Th17 cell frequency.

miRNA is a large class of non-coding single stranded RNA, which regulates about 1/3 of human genes and is essential in physiological processes such as cell growth, differentiation, immunity, and autoimmune disorders [9]. Several studies have shown that miRNA participates in the differentiation and development of Th17 cells. For example, miR-26a inhibited the production of Th17 cells by regulating IL-6 and was positively correlated with Foxp3 expression, promoting Treg cell development [16]. miR-301a also promotes differentiation of Th17 cells by targeting a inhibitory protein on STAT3-activated proteins [17]. The present study demonstrated that miR-153-5p was regulated by LINC-XIST. miR-153-3p inhibitor observably suppressed IL-17 concentration, mRNA expression of IL-17, and Th17 cell frequency while si-XIST reversed this impact. Thus, it can be seen that miR-153-5p improved Th17 cell differentiation, which was regulated via LINC-XIST.

In addition, ETS1 was found to be regulated by miR-153-5p. ETS1 is the most conserved protein in the ETS family. In young mice, ETS1 is highly expressed in various tissues [18]. In adult mice, ETS1 is mainly expressed in immune tissues [19]. There are many defects in the T cell lineage in ETS1 knockout mice, including abnormal thymus differentiation, decreased number of peripheral T cells and Treg cells, impaired function of Treg cells, and increased number of Th17 cells [20, 21]. There are also abnormalities in the process of B cell differentiation in ETS1 deficient mice, especially differentiation of B cells into plasma cells, which accumulate in peripheral lymphoid organs and bone marrow. The present study demonstrated that ETS1 was directly regulated via miR-153-5p. ETS1 observably suppressed IL-17 mRNA expression, IL-17 concentration, and Th17 cell frequency while miR-153-5p mimic reversed this impact. Thus, it can be seen that ETS1 suppressed Th17 cell differentiation, which was regulated via miR-153-5p.

In conclusion, LINC-XIST suppressed Th17 cell differentiation via targeting miR-153-3p/ETS1.

## Figures and Tables

**Figure 1:** Differentiation of Th17 cells. (a) IL-17 concentration was detected by ELISA. The expression of XIST (b) and miR-153-3p (c) was measured via qPCR. ^*∗*^*P* < 0.05.

**Figure 2:** XIST promoted Th17 cell differentiation. (a) The expression of XIST was measured via qPCR. (b) The mRNA expression of IL-17 was measured via qPCR. (c) IL-17 concentration was detected by ELISA. (d, e) The frequency of IL-17+ cells as a fraction of total CD4+ T cells was assessed by flow cytometry. ^*∗*^*P* < 0.05.

**Figure 3:** miR-153-5p was regulated by XIST. (a) Predicted binding sites. (b) miR-153-5p inhibited luciferase activity of XIST-WT. (c) The expression of miR-153-5p was measured via qPCR. ^*∗*^*P* < 0.05.

**Figure 4:** XIST reverses the promoting effect of miR-153-5p on Th17 cell differentiation. (a) The expression of miR-153-5p was measured via qPCR. (b) The mRNA expression of IL-17 was measured via qPCR. (c) IL-17 concentration was detected by ELISA. (d, e) The frequency of IL-17+ cells as a fraction of total CD4+ T cells was assessed by flow cytometry. ^*∗*^*P* < 0.05. I = miR-NC; II = miR-153-3p inhibitor; III = miR-153-3p inhibitor + si-NC; IV = miR-153-3p inhibitor + si-XIST.

**Figure 5:** miR-153-5p directly downregulated ETS1. (a) Predicted binding sites. (b) miR-153-5p inhibited luciferase activity of ETS1-WT. (c, d) The protein expression of ETS1 was measured via western blot. ^*∗*^*P* < 0.05.

**Figure 6:** miR-153-5p reverses the inhibiting effect of ETS1 on Th17 cell differentiation. (a) The mRNA expression of ETS1 was measured via qPCR. (b) The mRNA expression of IL-17 was measured via qPCR. (c) IL-17 concentration was detected by ELISA. (d, e) The frequency of IL-17+ cells as a fraction of total CD4+ T cells was assessed by flow cytometry. 1 = NC; 2 = ETS1; 3 = ETS1 + NC-mimic; 4 = ETS1 + miR-153-3p mimic. ^*∗*^*P* < 0.05.

## Data Availability

The data used to support the findings of this study are available from the corresponding author on reasonable request.
